# Human-Computer Interaction for Recognizing Speech Emotions Using Multilayer Perceptron Classifier

**DOI:** 10.1155/2022/6005446

**Published:** 2022-03-28

**Authors:** Abeer Ali Alnuaim, Mohammed Zakariah, Prashant Kumar Shukla, Aseel Alhadlaq, Wesam Atef Hatamleh, Hussam Tarazi, R. Sureshbabu, Rajnish Ratna

**Affiliations:** ^1^Department of Computer Science and Engineering, College of Applied Studies and Community Services, King Saud University, P.O. BOX 22459, Riyadh 11495, Saudi Arabia; ^2^College of Computer and Information Sciences, King Saud University, P.O. Box 51178, Riyadh 11543, Saudi Arabia; ^3^Department of Computer Science and Engineering, Koneru Lakshmaiah Education Foundation, Vaddeswaram, Guntur 522502, Andhra Pradesh, India; ^4^Department of Computer Science, College of Computer and Information Sciences, King Saud University, P.O. Box 51178, Riyadh 11543, Saudi Arabia; ^5^Department of Computer Science and Informatics, School of Engineering and Computer Science, Oakland University, Rochester Hills, MI 318 Meadow Brook Rd, Rochester, MI 48309, USA; ^6^Department of ECE, Kamaraj College of Engineering and Technology, Virudhunagar, TN, India; ^7^Gedu College of Business Studies, Royal University of Bhutan, Thimphu, Bhutan

## Abstract

Human-computer interaction (HCI) has seen a paradigm shift from textual or display-based control toward more intuitive control modalities such as voice, gesture, and mimicry. Particularly, speech has a great deal of information, conveying information about the speaker's inner condition and his/her aim and desire. While word analysis enables the speaker's request to be understood, other speech features disclose the speaker's mood, purpose, and motive. As a result, emotion recognition from speech has become critical in current human-computer interaction systems. Moreover, the findings of the several professions involved in emotion recognition are difficult to combine. Many sound analysis methods have been developed in the past. However, it was not possible to provide an emotional analysis of people in a live speech. Today, the development of artificial intelligence and the high performance of deep learning methods bring studies on live data to the fore. This study aims to detect emotions in the human voice using artificial intelligence methods. One of the most important requirements of artificial intelligence works is data. The Ryerson Audio-Visual Database of Emotional Speech and Song (RAVDESS) open-source dataset was used in the study. The RAVDESS dataset contains more than 2000 data recorded as speeches and songs by 24 actors. Data were collected for eight different moods from the actors. It was aimed at detecting eight different emotion classes, including neutral, calm, happy, sad, angry, fearful, disgusted, and surprised moods. The multilayer perceptron (MLP) classifier, a widely used supervised learning algorithm, was preferred for classification. The proposed model's performance was compared with that of similar studies, and the results were evaluated. An overall accuracy of 81% was obtained for classifying eight different emotions by using the proposed model on the RAVDESS dataset.

## 1. Introduction

Fewer emotions are critical in human-computer interaction [1]. Past years had increased interest in speech emotion recognition (SER), which uses speech cues to analyze emotion states. Nonetheless, SER remains a challenging endeavor due to extracting practical emotional elements. SER is handy for investigating human-computer identification. This indicates that the system must comprehend the user's feelings to define the system's activities appropriately. Numerous activities, including voice-to-text translation, feature extraction, feature selection, and classification of those characteristics to determine emotions, must be handled by a well-developed framework that incorporates all of these elements [2]. Classification of features is another problematic process requiring multiple emotional systems to execute the categorization correctly.

Speech contains two forms of information: textual and emotional. To achieve a harmonious human-computer interaction experience, the computer should automatically recognize the emotional content of voice signals. For example, the voice may gauge a client's emotions in a customer service system. It has been shown to increase children's social-emotional abilities and academic skills when used with an educational assistant system [3]. Parents and instructors are capable of resolving issues promptly. The operating system is capable of detecting emotions through speech. When the driver's mood is excessively nervous or furious, the system will provide an early warning. This may help lessen the likelihood of traffic accidents. Automatic speech emotion identification has a broad range of applications in various industries.

Emotion-oriented computing intends to automatically recognize and synthesize emotions expressed by speech, facial expression, or any other biological channel [4–6]. There is a wealth of research available on automated emotion identification in facial expressions [7–9]. Nevertheless, since emotion identification using face acknowledgment is computationally intensive, real-time implementation is impractical due to the need for high-quality cameras to capture facial photos. Apart from human facial expressions, language is a more promising mode of emotion identification. In addition, voice emotions play a significant role in multimodal human-computer contact [10, 11]. Therefore, language emotion detection is critical since voice is the primary medium of human communication. As a result, this article will discuss many features of speech emotion recognition (SER) approaches. The purpose of SER is to provide a sincere relationship.

By conversing with the machine using speech rather than conventional input methods, one can ensure that the machine understands the vocal content and more subtle indicators such as emotions, which any human hearer would readily respond to. If engines can understand emotional information, the link between man and machine will become more significant. SER evolved from a minor problem to a critical subject in human-computer interaction and speech processing during the previous decade. SER offers a broad range of possible uses. For instance, human-computer interfaces might be programmed to behave differently depending on the user's emotional state. This may be particularly critical in cases where voice is the dominant machine engagement [12]. As a result, SER is a necessary condition for humanizing the following apps and increasing their attractiveness among prospective users: robots [13], intelligent call centers, intelligent spoken teaching structures, intelligent aircraft cockpits, prosody for dialogue systems [14], ticket reservation systems, therapeutics, diagnostic tools, data mining for medical examination, in-car board structure [15], speech synthesis, computer games, voicemail filtering, intelligent toys, lie detectors, automatic research in films and television shows, and telephone banking, among other things.

The current work aims to develop a simple, efficient, and highly accurate model capable of classifying the emotions from speech data. In order to reach our goal, we have changed the state-of-the-art MLP designs. Because the training dataset was not supplemented to correct the imbalance between classes, it was possible to test the model's learning capacity with data limitations.

The list of contributions of the current work is as follows:

- A novel MLP network with the number of layers different from that of the state-of-art designs was designed.
- The usage of the adaptive learning rate instead of a constant one makes the model converge to optimum values.
- The model used the short-time Fourier transform and Mel-spectrum features.
- The model classified 8 different emotions with 81% accuracy on test data.
- The proposed model can achieve the desired results with fewer training data—there is no need to apply augmentation.
- The training time was quite short, a few minutes, since it is a simple model compared to state-of-the-art models.

The organization of the current paper is as follows: Section 2 of this study discusses prior efforts in the same topic. Sections 3 and 4 describes the dataset, the feature extraction process, the proposed algorithm, and the experimental design.  Section 5 discusses the performance and makes comparisons to previous works. The paper concludes with a conclusion in Section 5.

## 2. Literature Review

Cognitive psychologists' theories of emotions provide a valuable beginning point for demonstrating human feelings. While other theoretical models of emotion exist, the models employed most often are dimensional [16] and definite ones [17, 18]. Categorical representation of emotions has been increasingly utilized in affective computing for practical reasons. For instance, a previous study [19] implemented algorithms that distinguish eight distinct emotion types based on facial expressions. Oudeyer [20] created such algorithms to generate and identify five emotions using voice characteristics. According to Ekman and Friesen [13], six fundamental categorical emotions are universal, and their facial expressions are exhibited and recognized in all societies.

ML paradigms play a significant role in many papers on SER published in the literature [21]. Numerous articles detail the research conducted utilizing a variety of categorization approaches. In a previous study [22], support vector machines (SVMs) and decision trees (DTs) are related to identifying meaningful emotional states based on prosodic, disfluent, and lexical signals derived from practical oral human-human interactions. A previous study [23] also used the SVM approach to categorize emotional speech using two databases: Berlin German and Chinese. In another study [24], the authors built a hybrid system capable of recognizing people's emotions using their looks and speech information. Shami and Verhelst [25] explored three machine learning approaches—K-nearest neighbors (KNN), support vector machines (SVMs), and AdaBoost decision trees—and applied them to four emotional speech databases: Kismet, BabyEars, Danish, and Berlin. Rani et al. [26] conducted a comparative analysis of four machine learning (ML) techniques (KNN algorithm, regression trees (RTs), Bayesian networks, and SVMs) applied to the area of emotion identification utilizing physiological information. Another previous study [27] proposed a technique for recognizing human voice emotional conditions through a neural network classifier.

As with effective databases, most emotional dialogue acknowledgment systems are English-based. For languages like Basque and Spanish, techniques for voice recognition have been created, which are significantly less emotive. The study by Luengo et al. [28] is notable for Basque. Spanish literature includes works such as [29]. Another example is the work by Hozjan and Kacic [30], who investigated multilingual feeling identification in a variety of languages, including Spanish. 26 high-level (AHL) and 14 database-specific emotional (DSE) variables were employed in this study. AHL is the arithmetical depiction of low-level characteristics (low-level features are composed of pitch, pitch derivatives, energy, and a period of speech sections). DSE characteristics are a collection of speaker-specific emotional characteristics. Artificial neural networks were used to recognize emotions, and the max-correct assessment approach was used to acquire the findings. Identification using max-correct with AHL features was 55.21% on average, whereas identification using DSE characteristics was 45.76%. These assessed if cultural and linguistic differences affect emotional speech qualities. This component has been examined in several research studies, including [20], [31], and [32]. In [31], an experimental investigation was conducted comparing the Spanish and Swedish cultures. However, it should be noted that there is no reference in the literature to the Basque language being examined in the context of cross-cultural research on speech. In addition, a few everyday speech elements are presented in research using the Spanish language, and the majority of cross-cultural studies published in the literature are dependent on facial expression studies.

It is necessary to include Schroder's [33] study, which includes a lengthy bibliography of sources of emotional speech traits. The majority of these references are connected to English, and the characteristics cited by the writers are mostly seen in the literature. To the writers' knowledge, the study by Navas et al. [34] is exceptional in terms of emotional dialogue elements for Basque, and it also includes some of the most often seen traits. For Spanish, the state is similar; there are a few references, and some of the most prevalent elements are often utilized [24, 35]. On the other hand, a few previous studies [36 and 37] proposed a novel technique for signal processing that introduces new and fascinating elements for the analysis of voice emotion. Several works in the literature discuss feature extraction for emotion detection: [38] uses a fast correlation-based Filter to select the characteristics that will be used in a neural network classifier; [39] uses a professional to conduct the sampling; [40] uses a nonlinear dimensionality reduction to perform the recognition procedure; Picard et al. [41] presented and equated several procedures for feature-based recognition of the emotional state from this record.

There were also some recent works in the same domain with the recurrent neural networks along with the CNN. A recurrent neural network (RNN) can be used to infer associations from 3D spectrogram data across different timesteps and frequencies [42]. “Fusion-ConvBERT” is a parallel fusion model proposed by Lee et al. [43] that comprised bidirectional encoder representations derived from transformers and convolutional neural networks together. Zhang et al. [44] built a deep convolution neural network (DCNN) and a bidirectional long short-term memory with attention (BLSTMwA) model (DCNN-BLSTMwA) that can be utilized as a pretrained model for subsequent emotion recognition tasks.

## 3. Materials and Methods

### 3.1. The Dataset

The Ryerson Audio-Visual Database of Emotional Speech and Song (RAVDESS) dataset [45] originally contains 7356 files that include videos and audios of speeches and songs. Since our work is based on speech and the original dataset size is very large, which is 24.8 GB, it is decided to use the simplified version of the dataset on Kaggle [46]. This version of the dataset contains only speech data that are formatted as 16 bit, 48 kHz, .wav speech data files.

In this dataset, there are 1440 speech files that are prepared by 24 different actors, and their changers are also balanced as 12 males and 12 females. For each actor, there are 60 trials, so the total is 1440 files instead of 7356 files. In addition, the data size is decreased to 590 MB since there is only speech data audio instead of videos.

Song files are also included in our implementation to improve performance. Song contains fearful, sad, happy, calm, and angry emotions with 1012 files, where the song file of actor 18 does not exist. Therefore, the dataset contains 2452 audio files of emotions.

The dataset is created by 2 statements in a neutral North American accent to avoid the effects of words and focus more on emotions. These statements are “kids are talking by the door” and “dogs are sitting by the door”. In addition, the file names are coded with respect to identifiers, which are modality (audio, video, or both), vocal channel (speech or song), emotion, emotional intensity (strong or normal), statement (one of two statements), repetition (first or second) and actor (one of 24 actors; odd numbered ones are males). Some of the samples are displayed here wherein Figure 1 shows the audio sample for happy emotion, Figure 2 shows its spectrogram, Figure 3 shows the sad emotion audio file, and its spectrogram is shown in Figure 4. The speech emotions are classified as calm, happy, sad, angry, fearful, surprise, disgust, and neutral.

### 3.2. Preprocessing

To be able to perform preprocessing, data are investigated by data visualization methods. The balancing is checked, and the number of data is also checked. A sample from the data can be seen in Figure 5. The characteristics of the data are observed by using librosa library, which is commonly used to process audio data.

Then the number of speech data was also mentioned. However, this dataset also includes song data, which are also audio data. To increase the performance of the model, song data are also included during data preprocessing. Then the balance of the data was checked to see if there is any need to make a balancing process. The number of each sample for each class can be seen in Figure 6, and the numbers correspond to neutral, calm, happy, sad, angry, fearful, disgust, and surprised emotions, respectively. It can be also seen that the data are split by 25% as training and testing data.

Since there is no song file for actor 18, there is a balancing problem here; however, we did not perform any oversampling or undersampling operations here as we thought it was highly unnecessary, and we tried to challenge the model's capability. It was also possible to reduce the number of classes, which increases the performance; however, it was decided that the number of classes be 8.

### 3.3. Feature Extraction

For the feature extraction process, librosa, pandas, and NumPy libraries are used. To be able to apply the convolutional neural network, images of Mel spectrums are also obtained, but the results were not sufficient to process them. Instead of processing images of spectrums, one-dimensional features are extracted.

First, the mean of MFCC features is calculated; then short-time Fourier transform (STFT) and Mel spectrogram features are obtained by setting the sample rate of audio files, and the number of MFCC is set to 40. This process takes the longest time for all applications. Then, the obtained feature vectors are added sequentially and turned into a single vector. The vector that has 3 different properties is given as an input to the model.

### 3.4. MFCC

The first step in any speech recognition system is to extract features in order to be able to identify components of the audio signal that are good for identifying linguistic content and discarding other content carrying information such as background noise, emotion, etc. One of the most widely used feature extraction methods is the Mel-frequency cepstral coefficients method, shown in Figure 7. The audio path lies within the envelope of the short-term power spectrum. MFCCs occur to represent this envelope. MFCCs were introduced by Davis and Mermelstein in the 1980s for use in automatic speech and speaker recognition.

The Mel-frequency cepstrum is a representation of the short-term power spectrum of a sound based on a linear cosine transform of a log power spectrum on a nonlinear Mel-frequency scale. The Mel-frequency cepstral coefficients consist of a kind of cepstral representation of the audio clip. The main difference between the cepstrum and the Mel-frequency cepstrum is that in the MFC, the frequency bands are evenly spaced on the Mel scale, which approximates the response of the human auditory system closer to the linearly spaced frequency bands used in a normal spectrum.

### 3.5. Chroma Feature

Chroma features are an interesting and powerful representation of musical sound where the spectrums are projected into 12 different boxes representing the 12 different halftones of the musical octave. In music or speech phonics, chroma-based features, also called “pitch class profiles,” are a powerful tool for analyzing music and sound whose pitches can be meaningfully categorized. Chroma features are specifically aimed at representing the harmonic content of a short-lived sound window. Chroma features can show a high degree of robustness to changes in timbre and are closely related to the musical aspect of harmony. The various music processing tools are the chroma feature vector, chroma energy normalized statistics (CENS), constant-Q transform (CQT), short-time Fourier transform (STFT), etc. [47]

### 3.6. Model Architecture

The MLP is one of the most used and basic neural network architectures, and it can be also used for classification tasks. The MLP is also a supervised learning algorithm. A perceptron represents a one-neuron model, and a multilayer perceptron is a structure made of an input layer, hidden layers, and an output layer, as shown in Figure 8. It is a supervised learning algorithm that learns the function ^(^.^)^: Rm ⟶ R0 by training across a dataset. It is a nonlinear architecture for classification, or regression, given a set of *X*=*x*_1_, *x*_2_, *x*_3_,…*x*_*m*_ features and a target *y* corresponding to the data.

The input layer receives the data as input at the beginning, and then they are multiplied by weights to make the second layer, which is a hidden layer. Here, there are also activation functions that make the model learn nonlinear data. After the activation function operation, the calculation goes through the whole hidden layers until the last output layer. There are different types of activation functions such as the logistic activation function, hyperbolic tangent activation function, rectified linear unit activation function, etc. In our application, the rectified linear unit activation function is used. At the output layer, the size is defined by the number of classes.

The hidden layer is the next layer after the input layer, as shown in Figure 9. It is called the hidden layer because it is not exposed to direct input. The number of hidden layers created determines the depth of the model. As the number of hidden layers increases, the depth of the model increases. The rise of efficient libraries in computing power and developing technologies has allowed the creation of very deep neural networks.

If the last hidden layer is the output layer, it is called the output layer. It outputs a value or vector corresponding to the format required for the problem. Output can be determined by changing the output layer according to the problem. For example, for regression problems, the output may consist of a single neuron; for binary classification purposes, it may consist of 2 neurons; or for multiple classification problems, it may consist of more than one neuron.

At the end of the first feedforward operation, the error is estimated with respect to labels. The error function is called as the cost function, and there are different types of cost functions such as mean squared error, mean absolute error, and the cross entropy cost function. In this work, since the objective is classification, the cross entropy cost function is used. Then back propagation is performed to update weights, which is carried out by gradient descent. For this optimization, stochastic gradient descent is commonly used; however, for this work, an Adam optimizer is used. After training the model for some time and epochs, the model learns how to classify the data.

### 3.7. Evaluation Metrics

To understand how successful a classification problem or process is, we need to analyze our results with various evaluation criteria. In this study, F1-score, recall, precision, and accuracy metrics, which are the most widely used evaluation metrics, are preferred. These evaluation metrics are based on model prediction and actual data label attachment. By comparing these two situations, 4 different situations are formed:

- True positive: it is the case where data that the model predicts as True are actually True
- True negative: it is the case where data that the model predicts as False are actually False
- False positive: it is the case where data that the model predicts as False are actually True
- False negative: it is the case where data that the model predicts as True are actually False

The matrix created by the evaluation of the model on a set of data is called the confusion matrix, as shown in Table 1. Considering 4 different situations, accuracy, precision, recall, and F1-score metrics can be created. Each offers different information about model performance.

Accuracy can be briefly described as the ratio of all the correct answers (TP and TN) to all the answers, as shown in

(1) $$\begin{array}{c} Accuracy=\frac{TP+TN}{TP+TN+FP+FN}. \end{array}$$

Despite its frequent use, accuracy has a downside: it does not work well in unevenly distributed groups. Recall is the ratio of the positive classes (TP) we detected correctly to all positives (2). Precision is the ratio of the positive classes we detect correctly (TP) to all the data we label/name as true (TP + FP).

(2) $$\begin{array}{c} Recall=\frac{TP}{TP+FN}, \end{array}$$

(3) $$\begin{array}{c} \text{Precision}=\frac{\text{TP}}{\text{TP}+\text{FP}}. \end{array}$$

Increasing the Recall metric of our system in order to improve model performance may cause our Precision value to decrease. The important thing here is the priorities of your system. One needs to fine-tune this balance by analyzing the priorities. Another evaluation method that can be an alternative to Accuracy is the F1-score, which is more suitable to use for unbalanced distributed datasets. F1-score is the harmonic average of Precision and Recall. F1 penalizes the higher value, thus preventing it from manipulating the lower of the two higher values.

## 4. Results

For the training and testing parts, the data are split by 25% so that the performance can be checked on the data that were not seen by the model before. We could also perform the validation process here, but due to lack of data, several combinations are tried on separating them from training data by 20% to 30%; however, the validation data did not make a dramatic impact on test results; therefore, the data are just split as training and testing datasets.

To construct the model, the scikit-learn library and MLP classifier function are used. The activation function is selected as the rectified linear unit activation function, and an Adam optimizer is used. During the optimization, different types of optimizers, such as the stochastic gradient descent and quasi-Newton method (lbfgs), are used. In addition, different types of activation functions, such as the identity function, logistic sigmoid function, and hyperbolic tan function, are also used.

The shape of the hidden layer is set to 750 × 750 × 750, which makes the model a bit complex compared to its default layer size, which is only 100. However, due to this complexity, parameters for training are kept low, for example, the batch size is set to 128 and the maximum iteration number is set to 50. In addition, the learning rate is also optimized by setting the adaptive learning rate instead of the constant learning rate, which is the default application.

After setting the related parameters, training is applied on the model by the training dataset; it took just a few minutes to train the model, and the loss function graph can be seen in the figure.

As can be seen in Figure 10, the performance is quite well on training data, loss is decreased even after 20 iterations, and early stopping was used in case of nonincreased performance; however, since the loss kept getting lower, which cannot be seen in the figure due to small changes, the model stopped at the maximum iteration number.

Then, to be able to observe the performance of the MLP model, it is tested by the test dataset, which is not seen by the model during training. After applying the prediction, the confusion matrix below is observed.

From the confusion matrix in Figure 11 and the results for each emotion in Table 2, it can be easily said that the model is learned on the training dataset and performed well on the test dataset since it can distinguish most of the audio data with respect to 8 different classes. Since it is a bit hard to understand the model performance on each class, a classification report is used as in the table.

Table 3 shows that the overall accuracy reached 81% on average and the highest performance is observed on calm emotion while the lowest performance is observed on happy emotion.

## 5. Discussion and Comparison

Classification of emotions by only speech data is not an easy task even today; note that the number of emotions is eight for this dataset, which is quite high compared to the number of data that we have. Therefore, to obtain better results, it is always better to combine datasets and obtain a larger one and a more generalizable dataset to show better performance of the model. However, this work is focused on classifying these eight emotions and obtaining a sufficient result compared to existing works on this dataset.

The most challenging part of this task was to use this amount of data to train a model and perform the classification task for eight emotions. It gives much better results for a lower number of emotions; however, the challenge was to classify all these emotions. The model could perform well without any data augmentation, and we were also concerned that if it did, it would not converge properly, and hence, it would not yield superior results in the test dataset. As mentioned before, a better idea is to create a larger dataset and apply state-of-the-art models on it. However, even by using our simple model, we have reached high accuracy results.

### 5.1. Comparative Analysis

There exists a work which was carried out in 2021; it focused on combining several datasets (RAVDESS, TESS, and SAVEE) [47]. This is the application which we also suggest since the model becomes more generalized and is able to learn better. It also classified the same emotions and used MLP and convolutional neural network (CNN) models in it. Totally, it had 5732 unique voice files from these 3 different datasets, and it split their data as 25% for testing and 75% for training.

As a result of their application, it has reached 86.81% accuracy by using the CNN model and reached 83.32% accuracy by the MLP classifier. However, compared to our results, it is better, but we implemented it on a much smaller dataset. They also have their MLP classifier result by using only the RAVDESS dataset, and they reached 69.49% for eight emotions, which is quite low since we have reached 81% by using only the RAVDESS dataset (Table 4). They also tested their result on their CNN model, and the result is only 72.59%, which is also quite low compared to our result.

In addition, in another work that was published in 2021, they worked on improving the accuracy and robustness on IEMOCAP and RAVDESS datasets [51]. In their work, they proposed a method called head fusion to improve speech emotion recognition accuracy. They have proposed a new method that is based on multihead self-attention and used convolutional layers (attention-based convolutional neural network). As a result of their proposed method and experiments on IEMOCAP (interactive emotional dyadic motion capture) and RAVDESS datasets, they have reached 76.18% weighted accuracy and 76.36% unweighted accuracy. It can be seen that our result is better than that of this implementation since we have reached 81% accuracy (Table 4). However, they also injected 50 types of common noises, which is a different way of implementation and solving this task.  Figure 12 shows the confusion matrix of the proposed method on RAVDESS.  Table 5 indicates that the proposed model outperforms the already-mentioned previous works when we focus on each class of emotions separately.

## 6. Conclusions

This work is focused on improving the performance of a machine learning model in the speech dataset, which is the Ryerson Audio-Visual Database of Emotional Speech and Song. The dataset contains both speech and song data, with a total of 2452 audio files with 8 different emotions (calm, fearful, happy, surprise, sad, disgust, angry, and neutral emotions). The data are not balanced enough, but they are also not highly unbalanced. However, we did not perform any oversampling or undersampling operations on the data to see how well the proposed model will learn from the unbalanced data.

The most challenging part of this work was the lack of data, that is, why different types of approaches failed during training of a model such as decision trees, CNNs, random forests, etc. The best performance was obtained by the MLP classifier in previous works. Several parameters of a default MLP classifier are altered in this study, such as the design of the MLP classifier's hidden layer (750,750,750). Since the number of layers is quite high, it can cause overfit for high iteration rates; that is why the number of iterations during training is kept low so that overfitting is avoided. Otherwise, this model will cause overfit on training data for high iteration numbers on data-augmented datasets. For the preprocessing part, different approaches are also applied here. For CNN application, MFCC images are used but did not result in better performance, so the dataset is kept as a one-dimensional array. Feature extraction is the part that takes most of the time in this implementation, which took longer than that taken to train the model. The mean of MFCC features is calculated, and then short-time Fourier transform and Mel spectrogram features are obtained.

After the training process of the MLP classifier, the model is tested on the test dataset, which is 25% of the original data that was not used during training. As a result, an overall accuracy of 81% is obtained, whose performance is better than that of both the classification report and confusion matrix that was used. The highest performance is observed in calm emotion while the lowest performance is observed in happy emotion.

## Figures and Tables

**Figure 1:** Audio sample of happy emotion.

**Figure 2:** Spectrogram for an audio with happy emotion.

**Figure 3:** Audio sample of sad emotion.

**Figure 4:** Spectrogram for an audio with sad emotion.

**Figure 5:** Male happy speech data and its corresponding MFCC.

**Figure 6:** Training and testing data by 25% split.

**Figure 7:** MFCC extraction for happy sound data in RAVDESS dataset.

**Figure 8:** The basic structure of a multilayered perceptron [48].

**Figure 9:** One hidden layer MLP [49].

**Figure 10:** Training loss curve.

**Figure 11:** Confusion matrix for the test dataset (0: neutral, 1: calm, 2: happy, 3: sad, 4: angry, 5: fearful, 6: disgust, and 7: surprised).

**Figure 12:** Confusion matrix of the proposed method on RAVDESS [48].

**Table 1:** Confusion matrix.

True positive	False negative
False positive	True negative

**Table 2:** Confusion matrix of MLP classifier on RAVDESS [50].

Emotion	Angry	Calm	Disgust	Fearful	Happy	Neutral	Sad	Surprised
Angry	80.77	0.96	4.81	1.92	5.77	0.96	0.00	4.81
Calm	0.00	84.09	0.00	4.55	2.27	3.41	3.41	2.27
Disgust	7.84	3.92	50.98	3.92	1.96	3.92	5.88	21.57
Fearful	10.89	0.00	0.99	63.37	7.92	1.98	9.90	4.95
Happy	7.23	4.82	1.20	4.82	73.49	0.00	0.00	8.43
Neutral	0.00	11.11	0.00	3.70	1.85	64.81	9.26	9.26
Sad	1.03	11.34	2.06	13.40	3.09	1.03	59.79	8.25
Surprised	2.86	0.00	2.86	8.57	8.57	0.00	8.57	68.57

**Table 3:** Classification report of the prediction on test data.

	Precision	Recall	F1-score
Neutral	0.88	0.88	0.88
Calm	0.91	0.95	0.93
Happy	0.71	0.67	0.69
Sad	0.70	0.81	0.75
Angry	0.84	0.78	0.81
Fearful	0.87	0.85	0.86
Disgust	0.78	0.69	0.73
Surprised	0.71	0.77	0.74
Accuracy			0.81
Macroaverage	0.80	0.80	0.80
Weighted average	0.81	0.81	0.81

**Table 4:** Comparison of accuracy of the proposed work with that of previous works.

Models	Accuracy (%)
[50]	69.49
[51]	76.36
Proposed model	81

**Table 5:** Comparison of performance of the model on different emotions with previous works.

	Neutral (%)	Calm (%)	Happy (%)	Sad (%)	Angry (%)	Fearful (%)	Disgust (%)	Surprised (%)
[50]	64.81	84.09	73.49	59.79	80.77	63.37	50.98	68.57
[51]	65	71	70	81	88	89	73	81
Proposed	88.29	90.72	71.11	70.3	83.9	86.95	78.31	71.15

## Data Availability

The dataset used in this study can be accessed from “https://www.kaggle.com/uwrfkaggler/ravdess-emotional-speech-audio.”
